# Randomness for Nucleotide Sequences of SARS-CoV-2 and Its Related Subfamilies

**DOI:** 10.1155/2020/8819942

**Published:** 2020-11-14

**Authors:** Ray-Ming Chen

**Affiliations:** School of Mathematics and Statistics, Baise University, 21, No. 2 Road, Zhongshan, Guangxi Province, China

## Abstract

The origin and evolution of SARS-CoV-2 has been an important issue in tackling COVID-19. Research on these topics would enhance our knowledge of this virus and help us develop vaccines or predict its paths of mutations. There are many theoretical and clinical researches in this area. In this article, we devise a structural metric which directly measures the structural differences between any two nucleotide sequences. In order to explore the mechanisms of how the evolution works, we associate the nucleotide sequences of SARS-CoV-2 and its related families with the degrees of randomness. Since the distances between randomly generated nucleotide sequences are very concentrated around a mean with low variance, they are qualified as good candidates for the fundamental reference. Such reference could then be applied to measure the randomness of other Coronaviridae sequences. Our findings show that the relative randomness ratios are very consistent and concentrated. This result indicates their randomness is very stable and predictable. The findings also reveal the evolutional behaviours between the Coronaviridae and all its subfamilies.

## 1. Introduction

COVID-19 has a huge impact on all works of life. To develop stable and trustworthy vaccines [1, 2], one needs to track and analyse the properties of SARS-CoV-2, which couples with MERS-CoV [3] and SARS-CoV which are the subfamilies of betacoronavirus. Besides, one also needs to compare the properties of its related families: alphacoronavirus, deltacoronavirus, and gammacoronavirus [4]. In the Coronaviridae, betacoronavirus is the most deadly subfamily. In the category, SARS-CoV, MERS-CoV, and SARS-CoV-2 emerged in 2003, 2012, and 2019, respectively. To evaluate and analyse their properties, there are many genomic, clinical, statistical, and analytical tools available. Among all the theoretical or clinical research, genetical analysis provides a straightforward way to delve into the structures of Coronaviridae [5, 6]. There are some researchers focusing on geographic, demographic, and genomic analysis to extract some patterns of the viruses [7, 8]. Though the origin and evolution of these viruses was studied previously—for example, MERS-CoV [9] and SARS [10, 11]—there is still a long way to map out the interaction of these viruses. Currently, there are many theories or evidence about the mechanisms regulating the evolution and mutation of SARS-CoV-2 [12–14]. Nonetheless, a decisive solution to reveal such mechanisms still depends on further research and findings. In this article, we analyse their properties from the point of randomness, i.e., the degree of randomness of their nucleotide sequences. We devise a structural metric which would be applied in measuring the distances between all sorts of the Coronaviridae nucleotide sequences and the randomly generated nucleotide sequences. These distances could indicate how far the Coronaviridae is with respect to the random nucleotide sequences.

We utilise the data of coronavirus genomes from NCBI datasets [15]. Then, we measure the distances for each individual subfamily of the Coronaviridae. Our results show this structural metric is very suitable in revealing the properties of randomness. Hence, the relative distances between the random sequences are fairly stable and concentrated—this feature makes the concept of randomness feasible. From these settings, we could then calculate their relative randomness ratios (RRR) and extract our findings and results from RRR. The method to implement this notion is characterized in Section 3, and the results of the implementation are listed in Section 4, and the conclusions are reached in Section 5.

## 2. Theoretical Settings

In order to clearly measure the distances between structures, we devise a structural metric in this section—which would be applied in the latter sections.

For any vector $\vec{v}$, we use $\vec{v}\left(j\right)$ or ${\vec{v}}_{j}$ to denote its *j*th element and $|\vec{v}|$ to denote its length. We also use ${\left\|\vec{v}\right\|}_{E}$ to denote its Euclidean norm.

### 2.1. Common Finite Interval (CFI)

Let *AFS* denote the set of all the ascending finite sequences. Let $\vec{v}$,$\vec{w}\in$*AFS* be arbitrary. Define the greatest lower bound $lb\text{by}lb\left(\vec{v},\vec{w}\right)=\max\left\{\vec{v}\left[1\right],\vec{w}\left[1\right]\right\}$. Define the least upper bound $ub\text{by}ub\left(\vec{v},\vec{w}\right)=\min\left\{\vec{v}\left[|\vec{v}|\right],\vec{w}\left[|\vec{w}|\right]\right\}$. Let $\vec{v}\left[a,b\right]$ denote the subsequence of $\vec{v}$ whose elements lie between *a* and *b*. Let $\text{Set}\left(\vec{v}\right)$ denote the set of all the elements of $\vec{v}$. Let $\text{Union}\left(\vec{v},\vec{w}\right)=\text{Set}\left(\vec{v}\right)\cup \text{Set}\left(\vec{w}\right)$. Let finite *K*⊆*R* be arbitrary. Let Sort(*K*) ∈ FINI denote the vector by sorting all the elements in *K*. Define a difference operator Diff over finite vectors by $\text{Diff}\left(\vec{v}\right)=\left(v_{2}-v_{1},v_{3}-v_{2},\cdots ,v_{n}-v_{n-1}\right)$, where $n=|\vec{v}|$.

**Definition 1 .**

For any $\vec{v}$, any *a* < *b*, define $\vec{v}\left[a,b\right]$ by $\vec{v}\left[a,b\right]=\left\{k\in \text{Set}\left(\vec{v}\right),a\leq k\leq b\right\}$.

**Definition 2 .**

(common subsequence).

If $\vec{v}$,$\vec{w}\in$*AFS*, we define $\vec{v}\wedge \vec{w}$ by $\vec{v}\wedge \vec{w}=\text{Sort}\left(\text{Union}\left(\vec{v}\left[lb,ub\right],\vec{w}\left[lb,ub\right]\right)\right)$.

This serves as the common structure between two structures.

(1) $$\begin{array}{c} N_{1}=\left(\text{A},\text{C},\text{C},\text{T},\text{A},\text{C},\text{G},\text{T},\text{G},\text{A},\text{C},\text{T},\text{C},\text{C},\text{C},\text{T},\text{G},\text{G}\right),\\ N_{2}=\left(\text{C},\text{C},\text{C},\text{A},\text{A},\text{T},\text{C},\text{G},\text{T},\text{A},\text{G},\text{T},\text{T},\text{A},\text{G},\text{T},\text{C},\text{T},\text{A},\text{T},\text{A},\text{C},\text{T},\text{G}\right). \end{array}$$

**Definition 3 .**

(ascending finite sequences).

Let [*a*, *b*] < (where*a* < *b*) denote the set of all the ascending real vectors whose first element is *a* and last element is *b*. Let FINI be the union set of all [*a*, *b*] < forany*a* < *b*, i.e., FINI = ∪{[*a*, *b*]<:*a* < *b*, *a*, *b* ∈ *ℝ*}.

**Definition 4 .**

(structural metric).

Define a distance function *δ* over FINI by $\delta \left(\vec{v},\vec{w}\right)=\left({\left\|\vec{v}\right\|}_{E}+{\left\|\vec{w}\right\|}_{E}\right)/2-{\left\|\vec{v}\wedge \vec{w}\right\|}_{E}$.

**Claim 1 .**

*δ* is a metric on *AFS*.

**Proof**

It can be proved, according to Definition 4, by taking all the possible cases regarding their relations of intervals into consideration.

**Claim 2 .**

If *d*_1_, *d*_2_, ⋯, *d*_*n*_ is a set of metrics over a set *K*, then *d*(*a*, *b*) = ∑_*j*=1_^*n*^*α*_*j*_ · *d*_*j*_(*a*, *b*) is also a metric on *K*.

**Definition 5 .**

It follows immediately from the definitions of a metric.

**Example 1 .**

Suppose nucleotide sequence *N*_1_, *N*_2_ are given above.

Let *p*_*i*Q_ denote the position of nitrogenous base Q in the sequence *i*. Let *p*_12Q_ denote the position of common sequence o*fp*_1Q_ and *p*_2Q_. Then, the results are presented in Table 1. Let BASES = {^“^A^”^, ^“^C^”^, ^“^G^”^, ^“^T^”^}. Now we define *δ*(*N*_1_, *N*_2_) = [∑_Q∈Bases_*δ*_Q_(*p*_1Q_, *p*_2Q_)]/4 = 1/4 · [(∑_Q∈Bases_‖*p*_1Q_‖_*E*_ + ‖*p*_2Q_‖_*E*_)/2 − ‖*p*_12Q_‖_*E*_], where the last equality comes directly from Definition 4. Since $\delta_{\text{A}}\left(p_{1\text{A}},p_{2\text{A}}\right)=\left(\sqrt{41}+\sqrt{71}/2\right)-\sqrt{26}=2.32,$$\delta_{\text{C}}\left(p_{1\text{C}},p_{2\text{C}}\right)=\left(\sqrt{41}+\sqrt{143}/2\right)-\sqrt{33}=3.44,$$\delta_{\text{G}}\left(p_{1\text{G}},p_{2\text{G}}\right)=\left(\sqrt{69}+\sqrt{106}/2\right)-\sqrt{26}=4.20,$$\delta_{\text{T}}\left(p_{1\text{T}},p_{2\text{T}}\right)=\left(\sqrt{48}+\sqrt{45}/2\right)-\sqrt{24}=1.92.$ Therefore, *δ*(*N*_1_, *N*_2_) = (2.32 + 3.44 + 4.20 + 1.92)/4 = 2.97.

The weights are all predetermined 1/4 for each nitrogenous base. These values could also be adjusted according to professional judgement. For example, the weights could be decided by the relative frequencies of the bases.  Example 1 lays a foundation of our latter arithmetical calculation.

## 3. Methods

There are several steps for calculating the relative randomness ratios (RRR).

- Generate a set of 1000 random nucleotide sequences whose lengths are all fixed at 30000. The generated random (nucleotide) sequences are presented in Table 2
- Each sequence is regarded as a node. We then calculate the distance matrix for these nodes. This metric is a weighted metric consisting of 4 metrics which measure the structural distance with respect to each nitrogenous base. A concrete computation is shown in Example 1
- Some patterned nucleotide sequences are created and their distances with random sequences are calculated. These sequences are nonessential. They are generated only for comparative purposes. The created (followed by rules) nucleotide sequences and their distances are presented in Table 3
- The structural distances between SARS-CoV-2 nucleotide sequences and random ones are calculated. The results are presented in Table 4
- The structural distances between MERS-CoV nucleotide sequences and random ones are calculated. The results are presented in Table 5
- The structural distances between SARS nucleotide sequences and random ones are calculated. The results are presented in Table 6
- The structural distances between alphacoronavirus nucleotide sequences and random ones are calculated. The results are presented in Table 7
- The structural distances between deltacoronavirus nucleotide sequences and random ones are calculated. The results are presented in Table 8
- The structural distance between gammacoronavirus nucleotide sequences and random ones are calculated. The results are presented in Table 9
- RRR for each subfamily is calculated and the way to calculate it is explained in Section 4.2

## 4. Results

We use R program 4.0.2 (version) which in particular involves a package “Biostrings” to help us implement the theoretical setting. By the procedures mentioned in Section 3, we present the results in this section. We set the length of random nitrogenous base to be 30000, which is pretty much the length for SARS-CoV virus family. We also use R to sample 1000 samples (sequences) for our experiment (due to the capacity of our computers).

### 4.1. Experiment: Randomness of Nucleotide Sequences

Through Definition 4 and Example 1, we have the distance matrix as follows:

(2) $$\begin{array}{c} \begin{array}{c} s_{1}\\ s_{2}\\ \vdots \\ s_{999}\\ s_{1000} \end{array}\left(\begin{array}{ccccccccc} \overset{s_{1}}{0} & \overset{s_{2}}{129.8} & \overset{s_{3}}{131.0} & \overset{s_{4}}{130.3} & \overset{\cdots }{\cdots } & \overset{s_{997}}{129.9} & \overset{s_{998}}{131.8} & \overset{s_{997}}{131.0} & \overset{s_{1000}}{131.0}\\ 129.8 & 0 & 130.2 & 130.9 & \cdots & 130.5 & 132.0 & 131.0 & 131.5\\ \vdots & \vdots & \vdots & \vdots & \cdots & \vdots & \vdots & \vdots & \vdots \\ 131.0 & 131.0 & 130.5 & 130.7 & \cdots & 131.9 & 131.7 & 0 & 131.8\\ 131.0 & 130.5 & 131.0 & 130.6 & \cdots & 130.2 & 131.4 & 131.8 & 0 \end{array}\right) \end{array}$$

After removing the diagonal, we calculate some descriptive values for the 999∗999 elements: the minimum, maximum, mean, and standard derivation of the whole distance matrix. The minimum is 127.1 and the maximum is 134.7. The mean is 130.88 and the standard derivation is 0.83. Since the standard derivation is very small, the structural distance between any pair of random nucleotide sequences is highly concentrated around the mean—this is a good referential property for our further analysis. Now, let us demonstrate the distances between some patterned sequences with random sequences.

**Example 2 .**

Suppose A, C, G, T are bundled and repeated 7500 times with ∣*q*_1_ | = 3000; moreover, AA, CC, GG, TT are bundled and repeated 3750 times with ∣*q*_2_ | = 3000; finally, AACGAT (a pattern for the Fibonacci sequence *F*_*n*_ with mod operation, or *F*_*n*_ mod 4, where 1, 2, 3, and 4 are identified with “A”, “C”, “G”, and “T”, respectively) are bundled and repeated 5000 times with ∣*q*_3_ | = 3000 as shown in the following:

- *q*_1_ = (^“^A^”^, ^“^C^”^, ^“^G^”^, ^“^T^”^, ^“^A^”^, ^“^C^”^, ^“^G^”^, ^“^T^”^, ⋯, ^“^A^”^, ^“^C^”^, ^“^G^”^, ^“^T^”^)
- *q*_2_ = (^“^A^”^, ^“^A^”^, ^“^C^”^, ^“^C^”^, ^“^G^”^, ^“^G^”^, ^“^T^”^, ^“^T^”^, ⋯, ^“^G^”^, ^“^G^”^, ^“^T^”^, ^“^T^”^)
- *q*_3_ = (^“^A^”^, ^“^A^”^, ^“^C^”^, ^“^G^”^, ^“^A^”^, ^“^T^”^, ^“^A^”^, ^“^A^”^, ⋯, ^“^C^”^, ^“^G^”^, ^“^A^”^, ^“^T^”^)

The distances between each *q*_*j*_ and the random sequences are listed in Table 3.

The structural distances between patterned sequences and random ones obviously have different results in comparison with the random sequences.

### 4.2. Distance for Nucleotide Sequences

We import SARS-CoV-2 genomic codes and save them in S4DSC2 [15]. Since the size of S4DSC2 is too huge (4617), or {*s*_1_, *s*_2_, ⋯, *s*_4617_}, and could not be handled by our computer, we sample only 20 of them. The results are presented in Table 4, where column “Sequence” is the order of the sampled sequence in the data set; “Min” and “Max” are the minimal and maximal distance for the given sequence with the random sequences, respectively; “Mean” is the average distance between the given sequence and the random sequences; “Sd” is the standard derivation of such set of distances; “Mean rand” is the average distance of the distance matrix of random sequences; “RRR” is the relative randomness ration, which is the “Mean” over “Mean rand.” For the latter tables, meanings of the columns are the same; we will skip the wording. For MERS-CoV, the size of data downloaded is 530. We sample 20 of them randomly. The results are presented in Table 5. For SARS-CoV, the size of data downloaded is 10647. We sample 20 of them randomly. The results are presented in Table 6. For alphacoronavirus, the size of data downloaded and filtered is 1002. We sample 20 of them randomly. The results are presented in Table 7. For deltacoronavirus, the size of data downloaded and filtered is 149. We sample 20 of them randomly. The results are presented in Table 8. For gammacoronavirus, the size of data downloaded and filtered is 427. We sample 20 of them randomly. The results are presented in Table 9.

## 5. Conclusion

By observing all the results presented in the tables, we could reach the following statements:

- The structural distances between random (nucleotide) sequences are highly concentrated with low standard derivation. This feature justifies the referential role under structural metric
- The patterned nucleotide sequences have lower means and lower standard derivations in distances with random sequences
- The relative randomness ratios (RRR) for Coronaviridae, which lie between 1.01 and 1.08, are much close to complete randomness ratio (or 1) in comparison with the ones for patterned nucleotide sequence, which lie around 0.84 in our examples
- Overall, the randomness of betacoronavirus is higher than alphacoronavirus or deltacoronavirus, which in turn are higher than the structural distances between SARS-CoV-2 and random sequences. This could probably explain why the mutations of betacoronavirus are higher than other subfamilies
- In the betacoronavirus, the RRR of SARS-CoV-2 is almost fixed at 1.04. This indicates the mutations of SARS-CoV-2 are stabilized at this moment

These findings provide some insightful knowledge about the degree of structural randomness of SARS-CoV-2 and its related family. Linking this knowledge to other research results and findings would help us map out the dynamical structures and evolutions of these viruses.

## Figures and Tables

**Table 1:** Position, difference vectors, and norms: *N*_1_ and *N*_2_.

Name	Position (index)	Difference vector	Norm
*p*_1_A	(1, 5, 10)	(4, 5)	$\sqrt{41}$
*p*_1_C	(2, 3, 6,11,13,14,15)	(1, 3, 5, 2, 1, 1)	$\sqrt{41}$
*p*_1_G	(7, 9, 17, 18)	(2, 8, 1)	$\sqrt{69}$
*p*_1_T	(4, 8, 12, 16)	(4, 4, 4)	$\sqrt{48}$
*p*_2_A	(4, 5, 10,14,19,21)	(1, 5, 4, 5, 2)	$\sqrt{71}$
*p*_2_C	(1, 2, 3, 7, 17, 22)	(1, 1, 4,10,5)	$\sqrt{143}$
*p*_2_G	(8,11,15,24)	(3, 4, 9)	$\sqrt{106}$
*p*_2_T	(6, 9, 12,13,16,18,20,23)	(3, 3, 1, 3, 2, 2, 3)	$\sqrt{45}$
*p*_12_A	(4, 5, 10)	(1, 5)	$\sqrt{26}$
*p*_12_C	(2, 3, 6, 7, 11,13,14,15)	(1, 3, 1, 4, 2, 1, 1)	$\sqrt{33}$
*p*_12_G	(8, 9, 11,15,17,18)	(1, 2, 4, 2, 1)	$\sqrt{26}$
*p*_12_T	(6, 8, 9,12,13,16)	(2, 1, 3, 1, 3)	$\sqrt{24}$

**Table 2:** 1000 sampled random nitrogenous bases.

Samples	Random sequence	Length
*s*_1_	CCTTTCGTTGCTCAT ⋯ GTTTATGGTACGCAGC	30000
*s*_2_	TGAGTATCTGGATCC ⋯ GCCACATGGCCAGTCC	30000
⋮	⋮	⋮
*s*_999_	TCGAGTGTCGGACTC ⋯ ATCCGGAGTTCTCCGA	30000
*s*_1000_	TAATCCAAAACAATA ⋯ AGCCTTAGGTCCTATT	30000

**Table 3:** Distances between patterned sequences and random ones.

	[*s*_1_, *s*_2_, *s*_3_, ⋯, *s*_998_, *s*_999_, *s*_1000_]	Min	Max	Mean	Sd.
*q*_1_	[106.9,107.3,107.0, ⋯, 108.7,108.0,107.5]	105.6	109.6	107.4	0.62
*q*_2_	[114.7,114.1,114.2, ⋯, 115.2,115.1,114.8]	112.8	116.4	114.7	0.58
*q*_3_	[110.1,110.5,110.4, ⋯, 111.7,111.3,111.0]	108.9	113.1	110.7	0.62

**Table 4:** Distance and randomness ratio between SARS-CoV-2 and random sequences.

	Sequence	Length	Min	Max	Mean	Sd.	Mean rand	RRR
1	1589	29903	133.78	138.00	135.92	0.72	130.66	1.04
2	1772	29671	133.50	138.03	135.71	0.71	130.52	1.04
3	3834	29903	133.73	137.95	135.88	0.72	130.60	1.04
4	483	29798	133.73	137.92	135.85	0.72	130.58	1.04
5	1333	29869	133.94	137.92	135.84	0.72	130.63	1.04
6	4515	29862	133.94	137.92	135.84	0.72	130.67	1.04
7	4100	29846	133.72	137.94	135.85	0.72	130.66	1.04
8	1005	29855	133.68	137.91	135.82	0.72	130.70	1.04
9	1132	29743	133.70	137.92	135.85	0.72	130.62	1.04
10	4218	29857	133.35	137.93	135.68	0.72	130.50	1.04
11	3391	29835	133.73	137.96	135.88	0.72	130.65	1.04
12	2187	29816	133.41	137.89	135.74	0.70	130.62	1.04
13	2802	29782	133.48	137.64	135.73	0.69	130.61	1.04
14	1125	29726	133.39	137.81	135.76	0.70	130.55	1.04
15	1681	29903	133.72	137.92	135.85	0.72	130.59	1.04
16	3388	29834	133.72	138.00	135.91	0.72	130.57	1.04
17	3407	29834	133.41	138.10	135.70	0.70	130.50	1.04
18	2030	29835	133.77	137.99	135.91	0.72	130.53	1.04
19	1800	29827	133.75	137.94	135.88	0.72	130.75	1.04
20	2023	29808	133.77	137.99	135.91	0.72	130.65	1.04

**Table 5:** Distance and randomness ratio between MERS-CoV and random sequences.

	Sequence	Length	Min	Max	Mean	Sd.	Mean rand	RRR
1	394	30123	131.29	135.49	133.26	0.71	130.88	1.02
2	315	30123	131.16	135.40	133.22	0.73	130.90	1.02
3	324	30123	131.12	135.37	133.22	0.71	130.50	1.02
4	381	30123	130.59	135.05	132.91	0.69	131.07	1.01
5	46	30094	131.77	136.29	133.88	0.74	131.09	1.02
6	392	30123	130.34	135.47	133.06	0.69	130.93	1.02
7	282	30123	130.75	135.36	133.00	0.70	130.77	1.02
8	6	30081	131.26	135.40	133.24	0.71	131.10	1.02
9	210	30096	131.27	135.52	133.26	0.71	130.97	1.02
10	386	30123	131.28	135.30	133.23	0.71	130.88	1.02
11	484	30096	130.75	135.06	133.03	0.71	130.32	1.02
12	506	30118	130.84	135.24	133.03	0.71	131.07	1.01
13	241	30123	130.69	135.23	133.02	0.70	130.81	1.02
14	359	30123	130.87	135.24	133.05	0.71	130.88	1.02
15	209	30096	131.22	135.47	133.23	0.71	130.85	1.02
16	469	29455	130.35	135.42	133.07	0.69	130.82	1.02
17	59	29919	130.70	135.90	133.22	0.74	130.80	1.02
18	366	30123	130.77	134.99	133.00	0.70	130.93	1.02
19	354	30123	130.88	135.26	133.05	0.71	130.41	1.02
20	128	30118	130.79	135.39	133.03	0.70	130.78	1.02

**Table 6:** Distance and randomness ratio between SARS-CoV and random sequences.

	Sequence	Length	Min	Max	Mean	Sd.	Mean rand	RRR
1	10218	29849	130.21	134.75	132.30	0.71	130.22	1.02
2	7750	29782	130.20	134.79	132.30	0.71	130.12	1.02
3	6483	29782	129.81	134.56	132.22	0.73	130.15	1.02
4	805	29882	129.98	134.51	132.27	0.72	130.18	1.02
5	2660	29900	129.50	134.75	132.26	0.71	130.29	1.02
6	1856	29865	130.17	134.74	132.31	0.70	130.68	1.01
7	7126	29835	130.25	134.57	132.31	0.73	130.43	1.01
8	87	29767	130.14	134.69	132.23	0.71	130.61	1.01
9	3289	29882	130.32	134.66	132.31	0.72	130.43	1.01
10	5307	29868	130.22	134.54	132.29	0.73	130.18	1.02
11	9593	29858	130.17	134.55	132.21	0.72	130.43	1.01
12	8925	29867	130.02	134.50	132.19	0.72	130.03	1.02
13	6020	29836	130.17	134.55	132.21	0.72	130.29	1.01
14	7029	29769	130.03	134.48	132.20	0.72	130.07	1.02
15	4783	29860	130.18	134.55	132.21	0.72	130.27	1.01
16	1804	29902	130.15	134.71	132.24	0.71	130.12	1.02
17	6852	29842	130.13	134.70	132.24	0.71	130.43	1.01
18	2415	29812	130.01	134.30	132.18	0.72	130.07	1.02
19	681	29890	130.12	134.46	132.25	0.72	130.52	1.01
20	3075	29808	130.11	134.46	132.23	0.73	130.41	1.01

**Table 7:** Distance and randomness ratio between alphacoronavirus and random sequences.

	Sequence	Length	Min	Max	Mean	Sd.	Mean rand	RRR
1	328	27993	126.25	131.20	128.95	0.71	126.58	1.02
2	205	27998	133.48	138.02	136.05	0.69	125.78	1.08
3	881	28029	133.65	138.18	135.79	0.74	125.28	1.08
4	137	27410	130.80	135.79	133.18	0.73	129.76	1.03
5	4	29355	130.70	135.07	132.75	0.69	128.91	1.03
6	877	27516	130.02	134.36	131.92	0.72	127.54	1.03
7	739	28009	129.30	133.56	131.45	0.70	128.01	1.03
8	723	28029	129.84	134.29	131.87	0.72	127.80	1.03
9	615	27489	133.74	138.24	135.92	0.73	126.11	1.08
10	140	27413	133.70	138.41	135.99	0.70	125.35	1.08
11	529	28595	129.90	134.35	131.89	0.71	127.58	1.03
12	764	28173	128.37	132.50	130.34	0.71	126.47	1.03
13	36	29295	127.71	132.27	129.86	0.70	125.47	1.03
14	118	29357	129.94	134.27	131.98	0.69	127.77	1.03
15	917	27165	129.79	133.95	131.95	0.72	127.72	1.03
16	686	28038	132.14	136.16	134.10	0.69	129.04	1.04
17	547	28521	126.37	131.24	129.01	0.71	126.92	1.02
18	820	28038	125.67	130.34	127.76	0.71	124.56	1.03
19	393	27993	125.36	130.07	127.45	0.70	124.85	1.02
20	238	27998	125.45	130.13	127.55	0.70	124.63	1.02

**Table 8:** Distance and randomness ratio between deltacoronavirus and random sequences.

	Sequence	Length	Min	Max	Mean	Sd.	Mean rand	RRR
	16	25422	125.14	129.84	127.57	0.70	122.91	1.04
2	117	25393	125.22	129.71	127.22	0.71	122.84	1.04
3	91	25399	127.27	131.43	129.42	0.73	123.05	1.05
4	33	25422	123.34	128.16	125.41	0.71	123.02	1.02
5	116	25414	119.74	124.91	122.56	0.69	120.45	1.02
6	87	25413	119.90	124.63	122.44	0.70	120.41	1.02
7	63	25420	122.77	127.27	124.98	0.70	122.04	1.02
8	73	25406	121.12	125.58	123.49	0.71	121.71	1.01
9	65	25420	123.14	128.15	125.31	0.72	123.23	1.02
10	138	26227	123.57	128.48	125.89	0.72	122.02	1.03
11	120	25403	124.56	129.30	126.97	0.72	122.48	1.04
12	129	25424	127.75	132.35	129.91	0.72	122.31	1.06
13	90	25414	120.35	124.48	122.43	0.71	120.53	1.02
14	107	25422	120.46	124.58	122.35	0.70	120.46	1.02
15	22	25408	120.41	124.54	122.48	0.71	120.22	1.02
16	4	26552	120.23	124.43	122.38	0.71	120.48	1.02
17	29	25422	120.33	124.48	122.45	0.71	120.46	1.02
18	119	25413	120.32	124.48	122.43	0.71	120.22	1.02
19	34	25438	120.33	124.50	122.44	0.71	120.41	1.02
20	131	26487	120.39	124.53	122.48	0.71	120.55	1.02

**Table 9:** Distance and randomness ratio between gammacoronavirus and random sequences.

	Sequence	Length	Min	Max	Mean	Sd.	Mean rand	RRR
1	134	27676	131.36	135.84	133.55	0.72	125.93	1.06
2	339	27603	130.72	135.93	133.04	0.71	125.69	1.06
3	385	27733	130.77	135.76	133.14	0.74	125.04	1.06
4	384	27755	130.64	135.54	132.79	0.74	124.90	1.06
5	87	27691	131.14	135.36	133.28	0.72	125.41	1.06
6	267	27675	130.46	135.08	132.82	0.74	125.49	1.06
7	151	27388	130.27	134.91	132.76	0.72	125.59	1.06
8	37	27690	130.98	135.48	133.13	0.70	125.50	1.06
9	47	27616	131.93	136.30	133.94	0.72	125.73	1.07
10	137	27618	130.94	135.36	133.25	0.72	125.39	1.06
11	88	27630	130.89	135.31	133.09	0.71	125.63	1.06
12	42	27620	131.08	135.88	133.47	0.71	125.95	1.06
13	238	27685	131.33	135.72	133.46	0.73	125.47	1.06
14	317	27590	142.40	147.90	145.41	0.73	130.85	1.11
15	133	27617	130.66	135.16	132.98	0.71	125.82	1.06
16	278	27686	130.74	135.31	133.08	0.71	125.44	1.06
17	144	27682	132.28	136.87	134.46	0.72	125.82	1.07
18	241	27685	131.28	135.79	133.44	0.71	125.37	1.06
19	334	27474	130.71	135.07	132.67	0.71	125.63	1.06
20	378	27642	129.80	135.01	132.44	0.70	125.72	1.05

## Data Availability

The data are available from the author on reasonable request (https://www.ncbi.nlm.nih.gov/sars-cov-2/; https://www.ncbi.nlm.nih.gov/datasets/coronavirus/genomes/).
